The article "A Network Meta-Analysis of the Differences in Effectiveness and Safety between Nivolumab and Targeted Drug Therapy in Metastatic Renal Cell Carcinoma" was published in 2022. Journal: J Oncol.

# A Network Meta-Analysis of the Differences in Effectiveness and Safety between Nivolumab and Targeted Drug Therapy in Metastatic Renal Cell Carcinoma

**DOI:** 10.1155/2022/5805289

**Published:** 2022-03-28

**Authors:** Hongchen Qu, Zhongyi Mu, Kai Wang, Bin Hu

**Affiliations:** Cancer Hospital of China Medical University, Liaoning Cancer Hospital & Institute, Shenyang 110042, Liaoning Province, China

## Abstract

**Objective:**

Nivolumab plus other drugs have provided significant benefits in patients with metastatic renal cell carcinoma (mRCC), but most of the available comparisons were conducted with sunitinib, and differences in efficacy with targeted drugs were marginally reported. Thus, this study used a network meta-analysis to compare the difference in efficacy between nivolumab combination therapy and other targeted agents.

**Methods:**

In this systematic review and network meta-analysis, we searched PubMed, Embase, and Cochrane Library databases for randomized controlled trials (RCTs) with the time set from database establishment to December 10, 2021, using programmed death factor 1 (PD-1) inhibitors, nivolumab, and sunitinib in the treatment of mRCC. Progression-free survival (PFS), overall survival (OS), response rate (RR), and adverse events (AEs) were collated and analyzed using the gemtc package in the R language.

**Results:**

A total of ten studies satisfied the inclusion criteria, including 6568 RCC cases, 10 drugs, and 11 treatment protocols. The Ate_Axi protocol obtained similar PFS to the Niv_Cab protocol, which outperformed that of all other protocols. The Niv_Cab regimen showed better PFS benefits than the Niv_Ipi regimen (HR < 1, *P* < 0.05), and Niv_Ipi had superior PFS compared to the Ate, Eve, Paz, Sor, and Sun scheme. The regimens Cab, Niv_Cab, and Niv_Ipi were associated with the best PFS benefits, while Eve is the least favorable drug in terms of PFS. Niv_Cab showed better OS than Ate_Bev, Eve, Paz, Sor, and Sun. The patients given Ate_Bev, Eve, Paz, Sor, and Sun had inferior OS to those given Niv_Ipi. The Pem_Axi, Niv_Cab, and Niv_Ipi regimens had the best OS, and that of Eve is considered least promising. The Niv_Cab protocol showed significantly better RRs than the Eve, Paz, Sor, and Sun protocols, and the Ate_Bev, Eve, Paz, Sor, and Sun protocols presented superior RRs compared to the Niv_Ipi protocol. The Ate, Eve, and Niv_Ipi regimens had the lowest incidence of AEs, and the Sor regimen had the highest incidence of AEs.

**Conclusion:**

Among the targeted treatment options for mRCC, both Niv_Cab and Niv_Ipi yield better efficacy and safety in the treatment of mRCC, with Niv_Cab providing more survival benefit but with a less favorable safety profile.

## 1. Introduction

Renal cell carcinoma (RCC) is a highly malignant tumor of the urinary tract, originating from the urinary tubular epithelial system of the renal parenchyma and accounting for approximately 80%–90% of renal malignancies [1]. Approximately 25% of patients with RCC are associated with distant metastases at the time of diagnosis, and another approximately 20–50% of patients with limited RCC eventually develop metastatic RCC (mRCC). Localized renal cell carcinoma is treatable by surgery, but mRCC is insensitive to conventional radiotherapy. Thus, there exists an urgent need to develop more effective treatment modalities [2]. Targeted therapy is the main direction of mRCC research, where a range of drugs such as sunitinib, atezolizumab, axitinib, bevacizumab, and cabozantinib has been widely used in the treatment of mRCC [3, 4].

Programmed cell death protein-1 (PD-1) and its ligand (PD-L1) inhibitors are immune sentinel monoclonal antibodies, and PD-1/L1 immunotherapy has become an important treatment for cancers, such as lung cancer, melanoma, and lymphoma, and has received widespread attention in the treatment of mRCC [5]. Research has revealed that PD-1/PD-L1 both alone and in combination with targeted agents increased drug response rates and provided significant survival benefits for patients, with good tolerability [6]. Nivolumab is a type of PD-1 inhibitor, and the CheckMate 025 and CheckMate 214 studies comparing the difference in efficacy between nivolumab combined with cabozantinib and ibritumomab and sunitinib both achieved significant results, providing new options for the treatment of mRCC [7]. The CheckMate 9ER showed that nivolumab plus cabozantinib had significant benefits over sunitinib with respect to progression-free survival and overall survival in patients with previously untreated advanced RCC [8]. Nevertheless, given the relatively short history of nivolumab's use in clinical settings, the small number of relevant studies, and the sole comparison with that of sunitinib in terms of efficacy, its differences with other targeted drugs regarding efficacy and safety require further evaluation. Sunitinib is the first drug approved for the adjuvant treatment of mRCC patients, and its efficiency as a first-line agent for mRCC has been confirmed by multiple data. Its difference in efficacy with sunitinib is the main basis for judging the effectiveness of new drugs [9]. This study used a network meta-analysis to include randomized controlled clinical studies with sunitinib as the first-line treatment regimen for mRCC and to indirectly compare the differences in efficacy and safety between targeted therapeutic agents and nivolumab combination therapy, and the results are reported below.

## 2. Materials and Methods

### 2.1. Literature Search

A literature search was conducted on PubMed, Embase, and Cochrane Library, with the time set from database establishment to December 10, 2021, using the search terms of (sunitinib [Title/Abstract]) OR (nivolumab [Title/Abstract]) and (((((renal carcinoma[Title/Abstract]) OR (renal cancer[Title/Abstract]) OR (Kidney Cancer[Title/Abstract])) OR (carcinoma of kidney [Title/Abstract])) OR (renal cell carcinoma [Title/Abstract])) and the corresponding Chinese search terms. Languages were set to English and Chinese, and references of the included literature were searched and retrospectively added to potentially missing studies whenever possible.

### 2.2. Inclusion and Exclusion Criteria

#### 2.2.1. Inclusion Criteria

(1) Study type included randomized clinical trials (RCTs); (2) study subjects were pathologically diagnosed with metastatic kidney cancer and received no radiotherapy prior to randomization; (3) with the comparison of at least two first-line systemic therapies for mRCC, at least one of which was sunitinib or nivolumab; (3) study endpoints included one of the following items: overall survival (OS), progression-free survival (PFS), response rate (RR), and adverse events (AEs); and (4) study design was scientific and standardized, with clear grouping and interventions and complete documentation such as follow-up data.

#### 2.2.2. Exclusion Criteria

(1) Non-RCT studies; (2) with the inability to obtain relevant outcomes such as OS, PFS, and AEs; and (3) less than 40 patients included in a single group.

#### 2.2.3. Literature Screening

Retrieval of data was performed by two investigators, and literature management was conducted using EndNote. Duplicate literature was excluded and screened separately for initial screening at three tiers: article title, abstract, and full text, before deciding whether to include in this study against the above criteria. The quality assessment of the included literature was performed as per the Newcastle–Ottawa Scale, and the decision to include was made by a third investigator independently in case of disagreement between the two investigators.

### 2.3. Data Extraction

The following data were extracted by two independent investigators from the included articles: first author's name, year of publication, subject type, number of subjects, treatment, study design, PFS, OS, RR, AEs, and other outcomes. OS, PFS, RR, and AEs were used as the main measures for the network meta-analysis.

### 2.4. Statistical Analysis

PFS was defined as the time from randomization to first imaging progression or death from any cause, and OS was defined as the time from randomization to death from any cause. RR was the proportion of patients enrolled and randomly assigned who achieved complete remission (CR) or partial remission (PR) per the investigator's assessment. AEs were clinical adverse events that occurred during or after the course of drug treatment. A network meta-analysis was performed for each outcome using random- and fixed-effects models with a Bayesian approach for direct and indirect treatment comparisons, with sunitinib or nivolumab combination treatment as the comparison group. HR and 95% CI were used for PFS and OS data outcomes, and odds ratio (OR) was used for RR and AE data outcomes. The R software gemtc package was used for all data analyses, and differences were considered by statistical significance bounds at *P* < 0.05.

## 3. Results

### 3.1. Eligible Literature

Of 314 original papers retrieved by an electronic search, 256 papers were excluded after literature abstract reading and exclusion of case reports, abstracts, and reviews, and 58 papers were coarsely included. Following the reading of the full text, studies with duplicate reports, unspecified data, subgroup analyses, and post hoc analyses were ruled out, and the final 10 pieces of literature were recruited. Of the 10 included documents, 9 were two-arm studies and 1 was a three-arm study. The three-arm study was converted into two two-arm studies for analysis, and a total of 10 drugs with a total of 11 treatment regimens were incorporated. The flow of the document search is shown in Figure 1, the basic information of the literature is shown in Table 1, and the network relationship of the included studies is shown in Figure 2.

### 3.2. PFS Analysis

A network meta-analysis was performed on PFS data from all studies with I2 = 8%, using a fixed-effects model. As shown in Figure 3(a), the Ate_Bev, Ate_Axi, Cab, Niv_Cab, Niv_Ipi, and Pem_Axi schemes had significantly better PFS than Sun (all HR < 1, *P* < 0.05) and the Eve scheme had significantly poorer PFS compared to Sun (all HR > 1, *P* < 0.05). Ate, Paz, and Sor showed similar PFS to Sun. Figures 3(b) and 3(c) show indirect comparisons of the differences in PFS between the different treatment regimens with the Niv_Cab and Niv_Ipi regimens. As shown in Figure 3(b), the Ate_Axi regimen PFS was not significantly different from the Niv_Cab regimen, and the rest of the regimens had significantly inferior PFS to Niv_Cab (all HR > 1, *P* < 0.05). In Figure 3(c), the Niv_Cab scheme had significantly better PFS than the Niv_Ipi scheme (HR < 1, *P* < 0.05), and less promising PFS was observed in Ate, Eve, Paz, Sor, and Sun schemes compared to Niv_Ipi (all HR > 1, *P* < 0.05).  Figure 3(d) shows the maximum potential for optimal PFS benefit for Cab, Niv_Cab, and Niv_Ipi protocols.

### 3.3. OS Analysis

A network meta-analysis was performed on OS data from all studies with I2 = 14%, using a fixed-effects model. As shown in Figure 4(a), the OS of Niv_Cab, Niv_Ipi, and Pem_Axi regimens was significantly better than Sun (all HR < 1, *P* < 0.05) and the OS of other regimens did not differ significantly from Sun. Figures 4(b) and 4(c) show indirect comparisons of the differences in OS between different treatment regimens and Niv_Cab and Niv_Ipi regimens. As shown in Figure 4(b), the OS of Ate_Bev, Eve, Paz, Sor, and Sun schemes was significantly inferior to that of Niv_Cab (all HR > 1, *P* < 0.05), and the OS of the remaining schemes was not significantly different from that of Niv_Cab. As shown in Figure 4(c), the Ate_Bev, Eve, Paz, Sor, and Sun regimens had significantly poorer OS than Niv_Ipi (all HR > 1, *P* < 0.05), and the remaining regimens had no significant difference in OS from Niv_Cab.  Figure 4(d) demonstrates an optimal OS benefit for the Pem_Axi, Niv_Cab, and Niv_Ipi programs with the highest probability.

### 3.4. RR Analysis

A network meta-analysis was performed on RR data from all studies with I2 = 0.3%, using a fixed-effects model. As shown in Figure 5(a), the RR of Niv_Cab, Niv_Ipi, and Pem_Axi regimens was significantly better than Sun (all OR > 1, *P* < 0.05) and the RR of other regimens was not significantly different from Sun. Figures 5(b) and 5(c) show the indirect comparison of RR differences between different treatment regimens with Niv_Cab and Niv_Ipi regimens. As shown in Figure 5(b), Eve, Paz, Sor, and Sun regimens had significantly inferior RR to Niv_Cab (all OR < 1, *P* < 0.05), and the rest regimens were similar to Niv_Cab. As shown in Figure 5(c), Ate_Bev, Eve, Paz, Sor, and Sun scheme RRs were all significantly inferior to Niv_Ipi (all OR < 1, *P* < 0.05), and RRs of the rest of the schemes were similar to Niv_Cab.  Figure 5(d) reveals that Niv_Cab, Ave_Axi, and Cab programs yield the highest probability of an optimal RR.

### 3.5. AE Analysis

A review of the AE data revealed a 100% incidence of AEs in the control group in the Sor study, which was the treatment regimen with the highest incidence of AEs. A net meta-analysis of AE data from other studies with I2 = 4% was performed with a fixed-effects model. The AE incidence of Ate, Eve, Niv_Cab and Ate_Bev regimens was significantly lower than Sun (all OR < 1, *P* < 0.05), and the AEs of other regimens were not significantly different from Sun, as shown in Figure 6(a). Figures 6(b) and 6(c) show the indirect comparison of the differences between different treatment regimens and Niv_Cab and Niv_Ipi regimen AEs. There was a significantly lower incidence of AEs in Ate, Ate_Bev, Eve, and Niv_Ipi regimens compared to Niv_Cab (all HR > 1, *P* < 0.05), and the remaining regimen AEs were not significantly different from Niv_Cab, as shown in Figure 6(b). As shown in Figure 6(c), Ate_Axi, Cab, Niv_Cab, Paz, Pem_Axi, and Sun regimen AEs were significantly higher than Niv_Ipi (all HR > 1, *P* < 0.05), and the remaining regimen AEs were not significantly different from Niv_Ipi.  Figure 6(d) shows that the Ate, Eve, and Niv_Ipi regimens have the highest probability of having the lowest incidence of AEs.

## 4. Discussion

This study compared the difference in efficacy of first-line treatment regimens for mRCC with sunitinib and indirectly compared the difference in efficacy and safety of combination therapy with nivolumab using network meta-analysis. The CheckMate 214 study demonstrated that nivolumab plus ibritumomab (Niv_Ipi) had a median OS of 55.7 months compared with sunitinib of 38.4 months in patients with intermediate-risk prognostic factors and poor prognostic factors, in the primary endpoint population and in all randomized patients; Niv_Ipi delivered more OS benefits and significantly improved RR [16]. The CheckMate 9ER study showed a significant prolongation of PFS and OS and improved RR with nivolumab in combination with cabozantinib (Niv_Cab) compared with the first-line treatment of mRCC using Sun, providing a new first-line treatment option for this subset of patients [8]. In the present study, the differences in the efficacy and safety of Niv_Ipi and Niv_Cab were indirectly compared with nine other treatment regimens with a comprehensive evaluation of their efficacy and safety. Niv_Ipi and Niv_Cab are the two large-sample, multicenter RCTs in which nivolumab is currently used, and no studies have yet directly compared the efficacy differences between the two regimens. This study found that Niv_Cab provided significantly higher PFS and RR than Niv_Ipi but significantly elevated the incidence of AEs and that Niv_Cab was able to provide more survival benefit, but had a poor safety profile.

In the present study, the top three studies for the likelihood of maximum PFS benefit were Cab, Niv_Cab, and Niv_Ipi. Cab is a multitargeted small-molecule tyrosine kinase inhibitor that is effective against a wide range of cancers. Research has revealed that Cab has a median PFS and median OS of 8.6 months and 26.6 months, respectively, both significantly higher than sunitinib at 5.3 months and 21.2 months [17]. Herein, an indirect comparison revealed that Cab was slightly more probable than Niv_Cab and Niv_Ipi for maximal PFS benefit, but it had no significant advantage in improving OS and enhancing RR, and its AEs were significantly higher than those of Niv_Ipi. Moreover, the top three studies with the potential for maximum OS benefit were Pem_Axi, Niv_Cab, and Niv_Ipi. Pem_Axi, a humanized anti-PD-1 monoclonal antibody, is the first anti-PD-1 agent to improve overall survival and progression-free survival in the first-line treatment of renal cell carcinoma [18]. A prior study has shown that Pem_Axi yields a higher survival benefit and comparable safety profile when compared to Sun in the treatment of renal cancer [6]. Indirect comparisons in this study showed that the Pem_Axi regimen had a significantly higher RR, a significantly lower PFS benefit, and a significantly higher incidence of AEs compared to Niv_Cab, Niv_Cab, and Niv_Ipi. The top three studies with the best RR potentials herein were Niv_Cab, atezolizumab plus axitinib (Ave_Axi), and Cab. The results of this study found no significant difference in OS and RR of Ate_Axi regimen in comparison with Niv_Ipi, but the incidence of AEs was significantly higher than that of Niv_Ipi; its PFS benefit was significantly lower than that of Niv_Cab. Atezolizumab is a tumor immunotherapy monoclonal antibody that, unlike tumor immunotherapy against PD-1, can activate T cells by binding to PD-L1 protein on the surface of tumor cells and on the surface of tumor-infiltrating immune cells, blocking the binding of PD-L1 to PD-1 and B7.1 receptor and prompting the human immune system to recognize and attack tumor cells [19]. The results of this study confirm that Ate_Axi has a lower safety profile compared to Niv_Ipi and poorer effectiveness than Niv_Cab.

One of the limitations of our study was that we did not collect the data on patients' age, gender, and medical history. However, these variables were often comparable in RCTs. Future studies are needed to verify the findings in our study.

To sum up, among the targeted treatment options for mRCC, both Niv_Cab and Niv_Ipi yield better efficacy and safety in the treatment of mRCC, with Niv_Cab providing more survival benefit but with a less favorable safety profile.

## Figures and Tables

**Figure 1:** Study flow diagram.

**Figure 2:** Network diagram of enrolled studies.

**Figure 3:** Network meta-analysis of PFS: (a) PFS compared with Sun, (b) PFS compared with Niv_Cab, (c) PFS compared with Niv_Ipi, and (d) stacking sort diagram of PFS.

**Figure 4:** Network meta-analysis of OS: (a) OS compared with Sun, (b) OS compared with Niv_Cab, and (c) OS compared with Niv_Ipi, and (d) stacking sort diagram of OS.

**Figure 5:** Network meta-analysis of RR: (a) RR compared with Sun, (b) RR compared with Niv_Cab, and (c) RR compared with Niv_Ipi, and (d) stacking sort diagram of RR.

**Figure 6:** Network meta-analysis of AEs: (a) AEs compared with Sun, (b) AEs compared with Niv_Cab, and (c) AEs compared with Niv_Ipi, and (d) stacking sort diagram of AEs.

**Table 1:** Basic information of the enrolled literature.

Author	Year	Phase	Indication	Treatment	Control	*N* (T)	*N* (C)	Outcomes
Eichelberg [10]	2015	III	NCT00732914	Sorafenib	Sunitinib	182	183	PFS, OS, RR, AEs
Motzer [11]	2013	III	NCT00720941	Pazopanib	Sunitinib	557	553	PFS, OS, RR, AEs
Motzer [12]	2014	II	NCT00903175	Sunitinib	Everolimus	233	238	PFS, OS, RR, AEs
Motzer [13]	2019	I b	NCT02684006	Sunitinib	Avelumab + axitinib	444	442	PFS, OS, RR, AEs
Rini [6]	2019a	III	NCT02853331	Sunitinib	Pembrolizumab + axitinib	429	432	PFS, OS, RR, AEs
McDermott [14]	2018	II	NCT01984242	Sunitinib	Atezolizumab + bevacizumab	101	101	PFS, OS, RR, AEs
				Sunitinib	Atezolizumab	101	103	PFS, OS, RR, AEs
Rini [15]	2019b	III	NCT02420821	Sunitinib	Atezolizumab + bevacizumab	461	454	PFS, OS, RR, AEs
Motzer [16]	2020	III	NCT01835158	Nivolumab + ipilimumab	Sunitinib	425	422	PFS, OS, RR, AEs
Choueiri [8]	2021	III	NCT03141177	Nivolumab + cabozantinib	Sunitinib	323	328	PFS, OS, RR, AEs
Choueiri [17]	2018	II	NCT01835158	Cabozantinib	Sunitinib	79	78	PFS, OS, RR, AEs

## Data Availability

The datasets used during the present study are available from the corresponding author upon reasonable request.
